# Correlation between Collateral Compensation and Homocysteine Levels in Patients with Acute Cerebral Infarction after Intravenous Thrombolysis Based on Medical Big Data

This article has been retracted.

**DOI:** 10.1155/2022/8213895

**Published:** 2022-08-31

**Authors:** Xiaohui Zhao, Fang Li, Yanfang Hu, Shaojie Yuan, Tong Zhang, Yu Yang

**Affiliations:** ^1^Neurology Department, Xingtai People's Hospital, Xingtai, 054000 Hebei, China; ^2^Obstetrics Department, Xingtai People's Hospital, Xingtai, 054000 Hebei, China; ^3^Pre-Hospital Emergency Department, Xingtai People's Hospital, Xingtai, 054000 Hebei, China

## Abstract

Homocysteine is an amino acid present in plasma, which is an important intermediate product in the metabolism of methionine and cysteine. Acute cerebral infarction (CI) is called acute CI of stroke. It is one of the most common diseases in neurology and has a serious impact, affecting people's lives. This article is aimed at studying the effect of data mining algorithms based on medical big data and the improved apriori algorithm on the analysis of the correlation between collateral compensation and homocysteine levels in patients with acute CI. This article proposes that there are many factors in patients with acute CI, among which are collateral compensation and homocysteine levels that are not easily determined. From the data in the tables in the experiment of this article, it can be seen that the collateral circulation of patients with acute CI is 8%, and the collateral circulation of patients without acute CI is 35%. The results indicate that both collateral compensation and homocysteine levels affect patients with acute CI. The higher the homocysteine level, the greater the probability of acute CI, and the better the state of collateral circulation, the less likely it is to suffer from acute CI.

## 1. Introduction

Most of the symptoms of cerebral infarction are not the same; these symptoms are many mild, patients are easy to ignore. The treatment of cerebral infarction in the early stage and cerebral hemorrhage is different. For the disease to timely diagnosis and treatment, with the development of economy, people pay less and less attention to their physical fitness, so more and more people suffer from acute CI. Acute CI refers to the symptoms of neurological deficits caused by the occlusion of cerebrovascular and interruption of the cerebral blood flow, which makes the brain tissue unable to obtain sufficient nutrients. And most of the patients will have sequelae, which will affect the physical and mental health and quality of life of the patients and seriously reduce the quality of life. Symptoms of acute cerebral infarction may vary depending on the location and degree of embolism. Patients may have contralateral hemiplegia, hemianopia, slurred speech, limb movement disorders, sensory disorders, and unresponsiveness.

Under normal circumstances, homocysteine can be catabolized in the body, and the concentration is maintained at a low level. However, in daily life, due to primary and secondary reasons, the metabolism of homocysteine in blood will be affected, resulting in the accumulation of homocysteine concentration, which is referred to as high blood homocysteine. Among many diseases, acute CI has the highest fatality rate, which has caused hard to eliminate troubles to people's life safety. With the aging of the population, the incidence of CI is getting higher and higher. Compared with cerebral hemorrhage, CI accounts for a larger proportion, accounting for about 70-80%. In China, acute CI threatens people's health and many people suffer from it. Therefore, prevention and treatment of CI has become extremely important.

With the continuous development of society, people's lifestyles are also changing, and the incidence of CI is increasing year by year. Naess et al. studied the time course of neurological deficits in patients with acute CI admitted shortly after the onset. They compared patients who were admitted to the hospital within 3 hours of the onset of symptoms due to CI with continuous NIHSS scores if feasible and compared them with patients who did not receive thrombolytic therapy. The short term refers to the NIHSS score and the modified Rankin score 7 days after the onset of disease. The hyperacute phase refers to a small time period of 6 to 9 hours after the onset, the acute phase refers to a time period of 6 to 9 hours and a time period of 21 to 27 hours, and the subacute phase refers to a period of 6 to 9 hours after the onset. The results showed that 552 patients obtained continuous NIHSS scores within 3 hours after the onset of stroke, which was significantly improved. Their research shows that timely treatment of patients with early pain will be greatly improved [1]. Dong et al. found that there is a close relationship between serum resistin levels and acute CI (ACI). They extracted data from eligible subjects and finally found that patients with acute CI had higher serum resistin levels. Their experiment tells people that the serum resistin level is related to ACI, but their experiment is not compared with the control group [2]. Chen discovered that the development of information and communication technology can promote the development of medical undertakings. Its development is receiving attention from scholars. Finally, he also found that medical big data has had a huge impact on the medical industry, but he did not describe the impact [3]. Price and Cohen found that big data has become the universal slogan of medical innovation. Medical big data is expected to revolutionize medical behavior. However, big data brings great risks, including major issues related to patient privacy. Here, Price and Cohen stated that big data has brought a lot of problems to patients' privacy. Price and Cohen also stated that the most important consideration for health privacy and patient governance data and the way to deal with data violations is medical big data [4]. Traditional medical imaging technology is an important part of medical physics; it is an advanced technical means developed with the concepts and methods of physics and physical principles. Godinho et al. found that medical imaging is conducive to the development of medicine; even small medical institutions have conducted research on it. But traditional medical imaging is difficult to adapt to today's medical big data, so they proposed a new method and created a new type of medical database. Their method has been verified. However, the scholars did not specify what their method is and what are the advantages compared with traditional methods [5]. Zhang and Wang discovered that today's medical system has security problems and faces many challenges. In order to improve the working efficiency of today's medical system, they designed a safe medical system. This new type of medical system can allow patients to understand their own conditions and better prevent and treat diseases, but the scholar did not use experiments to prove the authenticity and reliability of this system [6]. Shanmugapriya and Kavitha found that big data analysis has been widely used in various industries and is highly concerned by people, especially in the medical industry. They believe that the combination of cloud computing and medical data can effectively protect patients' privacy and information security issues, and it is also conducive to improving the work efficiency of medical staff and reducing their pressure. They researched a key method that can double-protect the safety of patients, but their research does not have any data to explain, so the authenticity remains to be investigated [7]. Xu et al. found that data mining has attracted more and more attention in recent years. Their main research is how to prevent privacy leakage caused by data mining operations. They found that data mining would bring serious privacy leaks, so they started a series of studies. But the scholars did not give a specific solution, nor did they mention how to reduce the risk [8]. Through the experimental analysis of scholars, it can be seen that medical big data has been greatly developed in recent years, and it is widely used in the medical industry. Research on patients with acute CI after intravenous thrombolysis based on medical big data is very necessary. However, the flaw in the experiments of scholars is that they did not use the algorithms of medical big data to calculate, so as to get accurate conclusions.

The innovations of this article are as follows: (1) It introduces the theoretical knowledge of medical big data and acute CI and uses data mining algorithms to analyze how medical big data researches on the correlation between collateral compensation and homocysteine levels in patients with acute CI after intravenous thrombolysis. (2) It analyzes the apriori algorithm before and after the improvement and conduct experiments and analysis on groups with and without acute CI after intravenous thrombolysis; experiments have found that collateral circulation compensation and homocysteine levels have an impact on acute CI.

## 2. Data Mining and Apriori Algorithm Based on Medical Big Data

The cloud service mentioned at this stage is not only a kind of distributed computing but also the result of the hybrid evolution and jump of computer technologies such as distributed computing, utility computing, load balancing, parallel computing, network storage, hot backup redundancy, and virtualization. Cloud computing is a type of distributed computing, which refers to decomposing huge data computing processing programs into countless small programs through the network “cloud” and then processing and analyzing these small programs through a system composed of multiple servers to obtain results and returned to the user. Cloud computing helps to achieve more convenient development, while relying on its own advantages to support the information reform of the medical industry. In addition, cloud computing also helps expand the mining of medical big data and information-based medical systems [9]. Therefore, in the future, the integration of cloud computing and medical big data will be further deepened. Apriori algorithm is a frequent itemset algorithm for mining association rules, and one of the most influential algorithms for mining frequent itemsets of Boolean association rules. The core idea is to mine frequent itemsets through two stages: candidate set generation and plot downward closure detection.

The apriori algorithm is an iterative process, which looks very simple, but notice that there are two important steps in each iteration: superset generation and support rate counting. The apriori algorithm can play a role in finding strong association rules and can find the correlation between collateral circulation compensation and homocysteine levels in patients with acute CI. The integration of medical big data and cloud computing will be an important development direction at present and in the future, which will bring huge development and changes to the entire medical industry [10]. Cloud computing provides solutions for medical big data, and how to mine useful association rules from these medical big data is one of the most important research topics [11].

The medical big data era not only analyzes the development of the medical industry but also summarizes and predicts the development and trends of the entire medical field through “Internet+medical” [12]. The structure diagram of medical big data is shown in Figure 1.

As shown in Figure 1, how to make it better standardized, managed, and shared is a major topic of future medical big data research. In addition, some predictive work should be done in combination with clinical practice to give full play to the advantages of medical big data. The establishment of the medical big data life cycle is about the preparation of medical big data and the application of medical big data results [13].

A decision tree is a decision analysis method to obtain the probability that the expected value of the net present value is greater than or equal to zero by forming a decision tree based on the known probability of occurrence of various situations, to evaluate the project risk, and to judge its feasibility. In this data mining step, it is necessary to extract the function of the hidden mode from the data according to the characteristics of the data itself and select the corresponding algorithm. Optional methods include clustering, decision trees, neural networks, and association rules [14]. Every scholar focuses on analyzing data and mining from different angles [15]. The process of data mining is shown in Figure 2.

As shown in Figure 2, data mining refers to the process of searching for information hidden in a large amount of data through algorithms. Data mining is generally related to computer science and achieves the above goals through a number of methods such as statistics, online analytical processing, intelligence retrieval, machine learning, expert systems (relying on past rules of thumb), and pattern recognition. At present, there are various forms of data mining methods. Data mining continuously integrates knowledge, technology, and research results in various fields in the process of research and development. In various forms, data mining continuously integrates knowledge, technology, and research results in various fields in the process of research and development. Through the use of data mining, abnormal data can be found, and the basic laws, patterns, and knowledge hidden by these data can be clarified [16]. This is a data mining method completely different from statistical analysis methods.

### 2.1. Neural Network Algorithm Based on Data Mining

The artificial neural network, also referred to as neural network or connection model, is an algorithmic mathematical model that imitates the behavioral characteristics of the animal neural network and performs distributed parallel information processing. The neural network is a multilayer feedforward neural network through back propagation of training data, and it is also the most widely used neural network model [17].

As shown in Figure 3, the artificial neural network does not need to determine the mathematical equation of the mapping relationship between the input and output in advance, but only through its own training, learns certain rules, and obtains the result closest to the expected output value when the input value is given. As an intelligent information processing system, the core of the artificial neural network to realize its function is the algorithm. In the process of learning the BP neural network error return attribute algorithm, each neuron in the input layer receives external input information and sends it to each neuron in the hidden layer [18]. The hidden layer in the middle is the internal information conversion layer for processing information. The middle layer can be designed as a single hidden layer or multiple hidden layers according to the needs of changing information functions. During training, the BP neural network can automatically extract the “reasonable rules” between the output and output data through learning and adaptively memorize the learning content in the weights of the network. That is, the BP neural network has a high self-learning and self-adaptive ability.

1. Forward propagation input

The connection of each neuron of the neural network will have a weight. The structure diagram of the forward propagation input is shown in Figure 4.

As shown in Figure 4, given node *j* of the output layer or hidden layer, the net input *H*_*j*_ to node *j* is as follows:

(1) $$\begin{array}{c} H_{j}=\underset{i}{\sum }w_{ij}y_{i}+\theta_{j}, \end{array}$$

where *y*_*i*_ is the output of node *i* in the upper layer and*θ*_*j*_ is the bias of node *j*. This bias is also called the threshold.

Given the net input *H*_*j*_ of node *j*, the output *Y*_*j*_ of node *j* is as follows:

(2) $$\begin{array}{c} Y_{j}=\frac{1}{1+e^{-1}}. \end{array}$$

The Sigmoid function represents the activity of the neuron represented by the node.

(2) Backward propagation error

The error Err_*j*_ calculation formula is as follows:

(3) $$\begin{array}{c} {\text{Err}}_{j}=Y_{j}\left(1-Y_{j}\right)\left(T_{j}-Y_{j}\right). \end{array}$$

Among them, the actual output is represented by *Y*_*j*_ and the known target value of a given training sample is represented by *T*_*j*_.

The error of the hidden layer node is

(4) $$\begin{array}{c} \Delta W_{ij}=\left(1\right){\text{Err}}_{j}y_{j}. \end{array}$$

The change of Δ*W*_*ij*_ is Err_*j*_*y*_*j*_:

(5) $$\begin{array}{c} {\text{Err}}_{j}=Y_{j}\left(1-Y_{j}\right)\underset{k}{\sum }{\text{Err}}_{k}\omega_{kj}. \end{array}$$

Backpropagation training uses the gradient descent method to continuously find the most suitable set of weights. The offset is updated by the following formula, where Δ*θ*_*j*_ is the change in offset of *θ*_*j*_, which is

(6) $$\begin{array}{c} \Delta \theta_{j}=\left(0\right){\text{Err}}_{j}. \end{array}$$

When processing a tuple, the bias and weight will be updated, which is a method of instance update, but in fact, the increment of bias and weight can be accumulated into the variable. After all tuples are processed in training, the bias and weight can be updated. For example, this method is a periodic update method; one cycle represents the iteration of scanning one training sample.

### 2.2. Global Algorithm Model Based on Data Mining

Given a data set *P*(*x* ≠ *x*) consisting of *n* samples and *m* features, it is known that it contains *C* patterns and *X* label information. Many existing mutual information-based feature selection methods are as follows:

(7) $$\begin{array}{c} P\left(x\neq x\right)\geq \frac{H\left(y_{i}\left|x\right.\right)-1}{\log c}. \end{array}$$

The model is trained in the normal forward training criteria, minimizing the label prediction loss (for samples in the source domain) and the domain classification loss (for all samples). Gradient inversion ensures that the feature distributions on the two domains are similar. In formula (7), *y*_*i*_ is the decision based on feature (*y*_*i*_|*x*), and *P*(*x* ≠ *x*) ≥ (*H*(*y*_*i*_|*x*) − 1)/log*c* is the real category. The goal of classification is to minimize the error of label prediction. Since *H*(*y*_*i*_|*x*) is a fixed amount, the problem is transformed into a maximum value. Once the feature with higher mutual information with the category label is selected, the error probability of classification will be reduced. So intuitively, the goal of using mutual information to solve the feature selection problem can be seen as finding the *T* feature sets that have the greatest dependence on the label *x*, and the goal of feature selection derived from this is

(8) $$\begin{array}{c} W^{*}=\arg\max\left\{D\left(a,b\right)\right\},d=\left(1,2,3,\cdots n\right). \end{array}$$

The standard uses the average value of the sum of mutual information between each feature *a* and *b* categories to approximate the “maximum dependence” standard *W*^∗^ as

(9) $$\begin{array}{c} W^{*}=\arg\max\left\{V\left(a,b\right)\right\},V=\frac{1}{W}\underset{V\in W}{\sum }\left(a,b\right). \end{array}$$

Adding the “minimum redundancy” condition to select mutually exclusive features as

(10) $$\begin{array}{c} W^{*}=\arg\max\left\{\frac{1}{W}\underset{V\in W}{\sum }\left(a,b\right)-\frac{1}{W^{2}}\right\}. \end{array}$$

The intuitive understanding is that the amount of information about feature *b* obtained after observing feature *a* is equal to the amount of information about feature 4 obtained after observing variable *b*. That is, (1/*W*)∑_*V*∈*W*_(*a*, *b*). This symmetry is a good attribute in feature selection.

The *SU*(*A*, *B*) between random variables *a* and *b* is defined as

(11) $$\begin{array}{c} SU\left(A,B\right)=2\frac{I\left(A,B\right)}{H\left(A\right)+H\left(B\right)}. \end{array}$$

This paper can make a global decision by systematically taking maximizing mutual information as a global optimization problem and considering the relevance and redundancy of all features at the same time.

### 2.3. Apriori Algorithm Based on Medical Big Data

The previous apriori algorithm is as follows:

1. The performance of the algorithm is reduced
2. The cost of the algorithm is increased
3. The efficiency of the algorithm is reduced

The basic idea of the apriori algorithm based on the division idea is to divide the transaction database into certain blocks according to the data size, search for frequent itemsets in each small block, and optimize the number of local prepruning and comparisons in each division.

Dividing a large number of data sets into disjoint and equivalent blocks. In each part of the block, calculate the minimum support in each block according to the minimum support originally set. Then, in each data block, compare with the calculated local minimum support to obtain the local frequent itemset. Assuming that there are *N* blocks in total, the minimum support is min − sup, and the number of transactions in each block is *D*_*m*_ is

(12) $$\begin{array}{c} \sup=\min-\sup*D_{m}\left(m=1,2,3,\cdots ,n\right). \end{array}$$

Joining step: If there is an itemset *L*_1_[2] for frequent self-joining operation of *L*_1_[1] itemset, its connection condition is

(13) $$\begin{array}{c} \left(L_{1}\left[1\right]=L_{2}\left[1\right]\right)\wedge \left(L_{1}\left[2\right]=L_{2}\left[2\right]\right). \end{array}$$

According to the optimization strategy of the previous comparison times, the algorithm is optimized and finally combined with the Hadoop model; this improved algorithm idea is transplanted to the Hadoop platform for parallel realization.

The apriori algorithm is an algorithm commonly used to mine data association rules, which can discover frequently occurring data sets in the transaction database. The rules formed by these associations can help to identify certain behavioral characteristics, while collateral circulation compensation in acute CI patients is associated with homocysteine. Correlations between amino acid levels can be mined by the apriori algorithm. Assuming that the data size of the original database is *P*(*DB*), the data transaction records are *N*, and the time to obtain the candidate *L*_*K*_ itemsets is the time of the connection step. Then, the time complexity of the traditional apriori algorithm can be obtained as

(14) $$\begin{array}{c} P\left(DB\right)=\underset{K\geq 2}{\sum }\left(P\left(L_{K}*L_{K+1}\right)\right). \end{array}$$

The apriori algorithm is

(15) $$\begin{array}{c} \overset{K}{\underset{K=N}{\sum }}P=\underset{K\geq 2}{\sum }\left(P\left(L_{K}*L_{K}\right)+P\left(L_{K}*L_{K+1}\right)\right). \end{array}$$

Therefore, it can be seen that the transaction database is divided based on the idea of division, and the algorithm is improved on this basis, so that the algorithm can reduce the number of comparisons, accelerate the pruning speed of the data set, and the design idea of parallel processing of data, so that the task of generating the candidate itemset is shared by all nodes, which solves the bottleneck problem of the apriori algorithm.

### 2.4. An Apriori_Pbcm Algorithm in a Cloud Environment

Although the apriori algorithm realizes the idea of parallelization and avoids multiple scans of the global database, when the data size is relatively large, the data itself occupies a large space. This research proposes an improved algorithm based on a compressed matrix. It only needs to do the inner product of the vector between the columns of the matrix.

In order to reduce the data set occupying a large amount of space, the matrix is compressed and improved, and combined with the MapReduce model, an Apriori_PBCM algorithm under the cloud environment is proposed.

Suppose there is an arbitrary database *Q*_*ij*_, with such a mapping relationship: *I*_*j*_ ∈ *T*_*i*_, which is *f*(*I*_*j*_) ∈ *T*_*i*_, where *T* is the number of transactions, and *Q* is defined as

(16) $$\begin{array}{c} Q_{ij}=\left\{\begin{array}{c} 1,I_{j}\in T_{i},\\ 0,I_{J}\notin T_{i}. \end{array}\right. \end{array}$$

According to formula (16), the Boolean matrix can be constructed as follows: where each row represents a transaction, and each column represents an item, which is

(17) $$\begin{array}{c} {DB}_{m\times n}=\left(\begin{array}{c} n_{11},n_{12},\cdots ,n_{1n}\\ n_{21},n_{22},\cdots ,n_{2n}\\ n_{m1},n_{m2},\cdots ,n_{mn} \end{array}\right). \end{array}$$

Among them, *n*_*mn*_ represents the number of rows of the Boolean matrix and *DB*_*m*×*n*_ is the number of transactions that do not include duplicates.

Candidate 1-itemset supports count formula:

(18) $$\begin{array}{c} \text{Support}\_\text{count}\left(I_{j}\right)=\overset{p}{\underset{i=1}{\sum }}\left(u_{ij}*\text{UW}\right). \end{array}$$

Among them, *u*_*ij*_ represents the corresponding transaction weight and its value represents the number of repeated transactions.

Candidate 2-itemset support count formula:

(19) $$\begin{array}{c} \text{Support}\_\text{count}\left(I_{i},I_{j}\right)=\overset{p}{\underset{i=1}{\sum }}\left(u_{ij}\wedge u_{kj}*\text{UW}\right). \end{array}$$

Among them, UW represents the corresponding transaction weight.

Compressing the matrix, delete row vectors with transaction length less than or equal to *k* and column vectors corresponding to infrequent *k*-itemsets, readjust the matrix to obtain matrix Support_count, and finally delete infrequent *k* − 1 itemsets. The support count formula for the candidate *k*-items set is

(20) $$\begin{array}{c} \text{Support}\_\text{count}\left(I_{1},I_{2},\cdots I_{K}\right)=\overset{p}{\underset{I=1}{\sum }}\left(u_{i1}\wedge u_{i1}\cdots u_{iK}*\text{UW}\right). \end{array}$$

Among them, (*I*_1_, *I*_2_, ⋯*I*_*K*_) represents the corresponding transaction weight.

The improved apriori algorithm in this paper only needs to scan the database once to convert it into a Boolean matrix. In the future, when calculating the support count of the candidate itemset, it only needs to use the characteristics of the matrix to perform the inner product between the column vectors. Moreover, the matrix is compressed by adding a weight array in the algorithm, which greatly reduces duplicate data and compresses transactions to save storage space, and the algorithm optimizes the end conditions, reduces the number of iterations, and improves the efficiency of the algorithm.

## 3. Experiment and Analysis of the Influence of Collateral Circulation and Homocysteine Levels on Patients with Acute CI

### 3.1. The Correlation between Patients with Acute CI and Collateral Circulation

Cerebral collateral circulation refers to a potential anastomotic channel that stabilizes cerebral blood flow when the main intracranial blood vessels are severely narrowed. Cerebral collateral circulation can remove tiny embolisms through its own circulation, reduce infarct volume, and play an important role in preventing CI.

The purpose of this experiment is to observe the compensation characteristics of cerebral collateral circulation in patients with CI and to investigate the relationship between the degree of cerebral collateral circulation compensation and CI.

This article investigates and studies on patients with acute CI and groups without acute CI, as shown in Tables 1 and 2.

As shown in Tables 1 and 2, the cerebral artery collateral circulation state of the acute infarction group was significantly worse than the cerebral artery collateral circulation state of the non-CI group, and the cerebral artery collateral circulation state of the acute infarction group was 12%-16%. The collateral circulation status of cerebral arteries in the non-CI group was 28%-35%.

This article compares the degree of collateral circulation in different groups of people, as shown in Figure 5.

As shown in Figure 5, the collateral circulation is the vascular network formed between the proximal and distal branches of the main vessel. These vascular networks are inherent, usually in a static state, and do not function. The state of collateral circulation of different groups of people is divided into three states: very poor, fair, and relatively good. The state of cerebral artery collateral circulation in the nonacute infarction group from 2015 to 2019 seems to be relatively good, the worst cerebral artery collateral circulation state is also 10%, and the best is 43%; the collateral circulation status of the cerebral arteries in the acute infarction group from 2015 to 2019 seems to be very poor. The worst cerebral artery collateral circulation status is as high as 41%, and the best is only 13%; it can be seen that the collateral circulation has a great influence on CI, and the correlation is also strong, the better the collateral circulation, the more helpful it is to prevent CI.

In summary, there is a strong correlation between collateral circulation and CI. In clinical work, correct evaluation of the establishment of collateral circulation is not only to formulate treatment plans for individual patients with CI but also to evaluate the clinical conditions of patients with CI. Therefore, how to promote the rapid establishment of collateral circulation and clarify the influencing factors of collateral circulation has gradually become the target of CI treatment, and further research is needed.

### 3.2. Correlation between Patients with Acute CI and Homocysteine Levels

As a nontraditional risk factor, research on the relationship between acute CI and changes in homocysteine levels has attracted more and more attention in recent years. There is an independent correlation between the increase in homocysteine levels and the occurrence of acute CI. Homocysteine levels are considered to be an independent risk factor for acute CI.

This article compares the levels of homocysteine, folic acid, and vitamins between the two groups with acute CI and those without acute CI, as shown in Table 3.

As shown in Table 3, the homocysteine level of patients with acute CI is 23.43 l, and the homocysteine level of patients without acute CI is 15.67 l. It can be seen that people with higher homocysteine levels are more likely to suffer from acute CI.

This article investigates the levels of homocysteine, folic acid, and vitamins in the two groups with and without acute CI from 2016 to 2020, as shown in Figure 6.

As shown in Figure 6, homocysteine levels without acute CI rose from 12.4 in 2016 to 16 in 2020, almost unchanged; however, the level of homocysteine in patients with acute CI rose from 22.3 in 2016 to 26, an average of about 24. It can be seen that there is a strong correlation between acute CI and homocysteine.

In short, the homocysteine level of patients with acute CI is significantly higher than that of the population without acute CI, and there is a positive correlation between acute CI and homocysteine; there is a negative correlation between acute CI and vitamins; the correlation between acute CI and folic acid is very weak.

### 3.3. Improved Apriori Algorithm Simulation Experiment and Analysis

In this paper, the classic apriori algorithm and the improved apriori algorithm are simulated and analyzed. Because of the confidentiality of medical data and electronic medical records, data mining training data is now used for simulation.

This article first tests the comparison of the mining time between the classic apriori algorithm and the improved apriori algorithm under the same degree of support, as shown in Table 4.

It can be seen from Table 4 that when the two algorithms set the same support threshold, the mining time is basically the same, and the improved apriori algorithm does not improve the time performance. Because the introduction of interest is improved in the calculation part of mining association rules, and the main time complexity of the algorithm is to find frequent items, so in terms of time complexity, improving the apriori algorithm does not improve the performance.

Secondly, carry out simulation test on the mining association rules. By setting different degrees of support, the classic apriori algorithm, the improved apriori algorithm with an interest threshold of 1, and the improved apriori algorithm with an interest threshold of 2 are compared; the specific data is shown in Table 5.

As shown in Table 5, in practical applications, relevant experts can set an appropriate minimum interest threshold through experience, so that association rules that users are not interested in can be filtered out. The algorithm overcomes the shortcomings of the classic algorithm that may dig out invalid strong association rules and optimizes the algorithm.

This paper investigates and compares the performance accuracy of the apriori algorithm before and after the improvement, as shown in Figure 7.

As shown in Figure 7, it shows the comparison between the classic algorithm, the improved algorithm with the minimum interest threshold, and the improved algorithm with the minimum interest threshold under different minimum support thresholds. It can be clearly seen that the improved algorithm mines fewer association rules under the same minimum support threshold, and the number of association rules mined is inversely proportional to the set minimum interest threshold.

## 4. Discussion

Based on the analysis of medical big data, this article explored the method of correlation between collateral circulation compensation and homocysteine level in patients with acute CI after intravenous thrombolysis. This article studies the related theories of collateral circulation compensation and homocysteine levels, and discusses the improved apriori algorithm through experiments.

This article also makes reasonable use of the apriori algorithm based on medical big data. As the application range of apriori algorithm becomes larger and larger, its importance also increases. According to this calculation, it is necessary to study the correlation between collateral circulation compensation and homocysteine level in patients with acute CI after intravenous thrombolysis based on medical big data.

In this article, we can learn from experiments on the correlation between collateral compensation and homocysteine levels in patients with acute CI after intravenous thrombolysis: groups with better collateral circulation are less likely to suffer from acute CI, so acute CI is related to collateral circulation; patients with acute CI have higher homocysteine levels than the general population, and the correlation between the two is positively correlated.

## 5. Conclusions

This article explains the concepts of collateral compensation and homocysteine levels in patients with acute CI and big medical data, and based on medical big data, data mining method, neural network algorithm, and apriori algorithm before and after improvement are proposed. It is proved that the improved apriori algorithm is beneficial to study the correlation between collateral circulation compensation and homocysteine level in patients with acute CI. Since big data technology is a relatively cutting-edge field, given the author's limited level of professional knowledge, there will inevitably be some shortcomings in the research and improvement of algorithms. Especially with regard to the mining of medical data, due to the complexity and diversity of medical data structure and the limitations of nonprofessionals, there are still many issues that need to be further thought and studied in the algorithm research work. The experiment finally found that there is a strong correlation between collateral circulation compensation and homocysteine levels in patients with acute CI. There is still much room for research on how to prevent acute CI by intervening these two factors.

## Figures and Tables

**Figure 1:** Structure diagram of medical big data.

**Figure 2:** Data mining diagram.

**Figure 3:** BP neural network.

**Figure 4:** Structure diagram of forward propagation input.

**Figure 5:** The degree of collateral circulation in different populations.

**Figure 6:** Comparison of homocysteine levels, folic acid, and vitamin levels in different populations.

**Figure 7:** Performance accuracy of apriori algorithm before and after improvement.

**Table 1:** Cerebral artery collateral circulation status in the acute infarction group.

Project	Age	Gender	Collateral circulation
A	22-26	Male	16%
B	27-31	Female	15%
C	32-36	Male	8%
D	37-41	Female	9%
E	41-45	Male	12%
F	46-51	Female	13%

**Table 2:** Cerebral artery collateral circulation status in the non-CI group.

Project	Age	Gender	Collateral circulation
A	22-26	Male	32%
B	27-31	Female	35%
C	32-36	Male	30%
D	37-41	Female	29%
E	41-45	Male	28%
F	46-51	Female	33%

**Table 3:** Investigation and comparison of the levels of homocysteine, folic acid, and vitamins between the two groups.

	HCY (*μ*mol/l)	Folic acid (ng/ml)	Vitamins (pg/ml)
Not suffering from acute CI	15.67	5.67	445.65
Acute CI	23.43	5.85	354.78
Correlation	Positive correlation	Generally	Negative correlation

**Table 4:** Comparison of the mining time between the classic apriori algorithm and the improved apriori algorithm.

Support threshold	Confidence threshold	Classic apriori algorithm	Improved apriori algorithm
0.25	0.5	30	50
0.30	0.5	32	31
0.35	0.5	3.6	3.5
0.40	0.5	0.5	0.4
0.45	0.5	0.3	0.5

**Table 5:** Improved apriori algorithm with different interest degree thresholds.

Support threshold	Confidence threshold	Classic apriori algorithm	Improved apriori algorithm	
			1	2
0.25	0.5	54353	25423	12343
0.30	0.5	55355	23232	14213
0.35	0.5	4353	4324	53242
0.40	0.5	5432	4231	34242
0.45	0.5	41234	41234	45321

## Data Availability

No data were used to support this study.
